# An Autophagy-Related Gene-Based Prognostic Risk Signature for Hepatocellular Carcinoma: Construction and Validation

**DOI:** 10.1155/2021/5770228

**Published:** 2021-10-13

**Authors:** Rui Feng, Jian Li, Weiling Xuan, Hanbo Liu, Dexin Cheng, Guowei Wang

**Affiliations:** ^1^Department of International Medicine, Zhejiang Provincial People's Hospital, People's Hospital of Hangzhou Medical College, Hangzhou City, Zhejiang Province 310000, China; ^2^Department of Interventional Medicine, The Affiliated Hospital of Qingdao University, Qingdao City, Shandong Province 266000, China; ^3^Department of Radiology, Xixi Hospital of Hangzhou, Hangzhou City, Zhejiang Province 310000, China; ^4^Department of Vascular Surgery-Center for Vascular Intervention, Zhejiang Provincial People's Hospital, People's Hospital of Hangzhou Medical College, Hangzhou City, Zhejiang Province 310000, China

## Abstract

**Background:**

Hepatocellular carcinoma (HCC) is a prevalent primary liver cancer. Treatment is dramatically difficult due to its high complexity and poor prognosis. Due to the disclosed dual functions of autophagy in cancer development, understanding autophagy-related genes devotes into novel biomarkers for HCC.

**Methods:**

Differential expression of genes in normal and tumor groups was analyzed to acquire autophagy-related genes in HCC. These genes were subjected to GO and KEGG pathway analyses. Genes were then screened by univariate regression analysis. The screened genes were subjected to multivariate Cox regression analysis to build a prognostic model. The model was validated by the ICGC validation set.

**Results:**

To sum up, 42 differential genes relevant to autophagy were screened by differential expression analysis. Enrichment analysis showed that they were mainly enriched in pathways including regulation of autophagy and cell apoptosis. Genes were screened by univariate analysis and multivariate Cox regression analysis to build a prognostic model. The model constituted 6 feature genes: EIF2S1, BIRC5, SQSTM1, ATG7, HDAC1, and FKBP1A. Validation confirmed the accuracy and independence of this model in predicting the HCC patient's prognosis.

**Conclusion:**

A total of 6 feature genes were identified to build a prognostic risk model. This model is conducive to investigating interplay between autophagy-related genes and HCC prognosis.

## 1. Introduction

Hepatocellular carcinoma (HCC) is a multistep and complex disease involved in epigenetic and genetic alterations, including genomic insertion, mutation, and deletion [1]. So far, certain therapeutic strategies like radical excision, liver transplantation, radiofrequency ablation (RFA), and arterial embolization (TAE) are expected to be applied in the treatment of this lethal disease [2–4]. Due to early diagnosis, intervention therapy, and development of therapies and surgery, the treatment for this cancer has been progressed greatly. However, most patients are diagnosed in the advanced stage due to lack of available biomarkers [5, 6]. Thus, there is an urgent need to decipher in-depth the pathways and mechanism of HCC progression.

Autophagy is a basic process to deliver damaged organelles and misfolded proteins to lysosomes for degradation to main intracellular homeostasis [7]. This process is involved in degeneration of dysfunctional cells [8]. Moreover, autophagy is also relevant to pathological process of liver injury and HCC [9, 10]. Thus, we thought that autophagy-related genes may participate in regulation of HCC or even most cancer development.

Due to rapid advancement in the high-throughput RNA profile, accessible gene expression data has been applied widely for cancer research. Extracting differently expressed genes by comparing tumor and normal tissues, followed by in-depth bioinformatics analyses for constructing prediction model, is a prevalent strategy. Based on the strategy, an emerging number of studies have proposed the HCC prognostic prediction model. However, for the practical application of the model, it is still needed to enhance the performance [11].

This investigation acquired the clinical data as well as expression data HCC and autophagy-related genes from bioinformatics databases. Autophagy-related genes in HCC were acquired through differential expression analysis. A prognostic model was built and validated through regression analyses. Altogether, a 6-gene-based prognostic risk model was determined. The model offers a candidate prognostic prediction strategy for HCC postoperation.

## 2. Materials and Methods

### 2.1. Data Preprocessing and Differential Expression Analysis

Firstly, mRNA expression data (normal: 50, tumor: 374) and corresponding clinical data (Supplementary Table 1) in the TCGA-Liver Hepatocellular Carcinoma (LIHC) dataset were downloaded. Then, 222 autophagy-related genes were accessed from the Human Autophagy Database (http://www.autophagy.lu/) (Supplementary Table 2). The expression of these genes was extracted from mRNA expression data in TCGA-LIHC. Differential expression analysis (∣logFC | >1, FDR < 0.05) was undertaken on the normal group and the tumor group using the “limma” package [12]. Differentially expressed autophagy-related genes were therefore obtained. Clinical data (like survival status and time) in Liver Cancer-RIKEN, Japan (LIRI-JP) were accessed from the International Cancer Genome Consortium (ICGC) (https://icgc.org/) as the validation set (Supplementary Table 3) to validate the multivariate prognostic model.

### 2.2. Gene Ontology (GO) and Kyoto Encyclopedia of Genes and Genomes (KEGG)

GO and KEGG enrichment analyses were conducted on the above autophagy-related genes in LIHC using the “clusterProfiler” package [13]. The “digest” and “GOplot” packages were applied for visualization.

### 2.3. Construction and Validation of a Prognostic Prediction Model

Univariate regression analysis was undertaken on differentially expressed genes (DEGs) using the “survival” package (*p* < 0.0001) [14]. Next, multivariate regression analysis was undertaken on the above screened genes using the “survival” package for establishment of a prognostic risk model. The patient's risk score was calculated according to the expression level of each gene. The median value of the risk score was deemed as a cut-off to distinguish high-risk and low-risk groups. Patient's survival curve was drawn by the “survival” package. The R package “survivalROC” was used to draw 3-year and 5-year OS receiver operating characteristic (ROC) curves. The area under the curve (AUC) was calculated.

### 2.4. Validation of the Risk Model with Clinical Information

We validated to assure whether the predictive performance of the model was independent of other clinical variables (including age, sex, T stage, and clinical stages). Univariate and multivariate Cox regression analyses were undertaken on clinical data in TCGA-LIHC as well as risk score. ROC curves of clinical characteristics and risk score were drawn.

### 2.5. Drawing and Validation of the Nomogram

A nomogram was established with clinical information and risk score to predict the possibility of 3-year and 5-year OS of HCC patients. Effectiveness of the nomogram was evaluated by the calibration curve.

## 3. Results

### 3.1. Data Preprocessing and Differential Expression Analysis

mRNA expression data and autophagy-related genes were first obtained. Afterwards, the “limma” R package was applied to determine DEGs from TCGA-LIHC, which was then overlapped with autophagy-related genes for obtaining autophagy-related DEGs. Altogether, 42 autophagy-related DEGs in LIHC were found (upregulated: 37; downregulated: 5) (Figure 1(a)). A boxplot of the expression of these genes in samples is shown in Figure 1(b).

### 3.2. Enrichment Analysis of Autophagy-Related DEGs

Some basic signaling transduction pathways and biological processes regulated by autophagy-related DEGs in HCC were further analyzed. Enrichment analyses were undertaken on 42 obtained DEGs. GO enrichment analysis revealed the main enrichment of DEGs in the regulation of autophagy, neuronal death, regulation of apoptotic signaling pathway, and that sort of biological processes (Figure 2(a)). KEGG illuminated that DEGs were mostly enriched in cellular senescence, cell apoptosis, and PI3K-Akt signaling pathways (Figure 2(b)).

### 3.3. Construction and Validation of a Model

Univariate regression analysis was undertaken on autophagy-related DEGs based on TCGA-LIHC (training set) (*p* < 0.0001). 21 genes remarkably relevant to patient's prognosis were obtained to draw a frost plot (Figure 3(a)). Genes were screened by multivariate regression analysis to establish the model. Finally, a 6-gene-based prognostic risk model was determined (Figure 3(b)). LIHC patients were classified into low- and high-risk groups. A risk score distribution plot (Figure 3(c)) and survival status plot (Figure 3(d)) were obtained. Moreover, the drawn ROC curves exhibited that AUC values of 5-year and 3-year OS were 0.733 and 0.717, respectively, (Figure 3(e)). The Kaplan-Meier cumulative curve suggested that the low-risk score patients had remarkably longer OS (Figure 3(f)).

Universality of the model was validated by the ICGC validation set LIRI-JP. AUC values of 5-year and 3-year OS were, respectively, 0.772 and 0.822 (Figure 3(g)). Survival curves showed a longer survival of patients a having low-risk score (Figure 3(h)). Taken together, the model held high accuracy.

### 3.4. Validation of the Independence of the Risk Model with Clinical Data

Risk score, clinical stages, and T stage all showed significant influence on the patient's prognosis (Figure 4(a)), while the multivariate regression analysis exhibited that only the risk score held a significant effect on patient's prognosis (Figure 4(b)). ROC curves based on clinical characteristics and risk score showed that AUC of risk score (0.78) was higher than that of all clinical characteristics (Figure 4(c)). Of all of the above, the prognostic model was a favorable prognostic prediction indicator which was better than the patient's clinical characteristics and independent from clinical characteristics themselves.

### 3.5. Drawing and Validation of the Nomogram

The nomogram has been widely employed in predicting a cancer patient's prognosis. It is mainly because it can simplify the statistical prediction model into a single value evaluation of the individual's OS possibility. The nomogram generated by clinical characteristics (T stage, sex, age, and clinical stages) and risk score could be used to predict OS of HCC patients (Figure 5(a)). Performance of the nomogram was predicted by calibration curves, and a high fitting level was observed (Figures 5(b) and 5(c)). On the whole, the nomogram is capable of accurately predicting the patient's prognosis, fueling an opportunity for the following consultation, decision, and arrangement.

## 4. Discussion

HCC is a global health concern on cancer. Its complexity and poor prognosis preclude effective access to treatment. Finding helpful biomarkers and constructing robust prognostic models to predict patients' prognosis are of general interest for HCC therapy.

Biomarkers for HCC diagnosis and prognosis have been screened in the past few decades, and several prognostic prediction models were constructed. A risk model was established based on 7 autophagy-related genes (SPHK1, HSPB8, ITGA3, CDKN2A, BIRC5, IKBKE, and TMEM74) in HCC (Wang et al. [15]). Potential core genes associated with HCC progression and prognosis were identified by bioinformatics analysis: CCNB1, CCNA2, CCNB2, NCAPG, PBK, NUSAP1, AURKA, ZWINT, PRC1, and KIF4A (Song et al. [16]). This paper identified 6 gene signatures (EIF2S1, BIRC5, SQSTM1, ATG7, HDAC1, and FKBP1A) by differential expression analysis, univariate analysis, and multivariate analysis in TCGA-LIHC. These autophagy-associated DEGs in HCC were used to build a prognostic prediction risk model. Compared with the previous studies focusing on autophagy-associated prognostic signature [17–19], our model presented an advantage with the relatively higher risk score (about 1.5) and reliable *p* value. To sum up, our results provide a novel perspective for precise prediction of HCC prognosis.

Regulation of these 6 genes were proven in assorted cancers except HCC. Sequestosome 1 (SQSTM1) encodes a multifunctional protein that binds to ubiquitin. p62 was confirmed to inhibit autophagy flux and promote epithelial-mesenchymal transformation in metastatic prostate cancer by maintaining the level of HDAC6 [20]. Sequestosome 1 is an effective prognostic factor associated with cell proliferation in human colorectal cancer [21]. In addition, p62 is upregulated in the prophase of HCC and induces cancer by maintaining the survival of stress-induced HCC-initiating cells [22]. HDAC1 mediates eukaryotic gene expression. It has been reported to promote glycolysis in gastric cancer, and it is an independent adverse prognostic factor for disease-free survival and OS [23]. Silencing of HDAC1 enhances the sensitivity of ovarian cancer to chemotherapy [24]. HDAC1 restrains Snail2-mediated epithelial-mesenchymal transition (EMT) in the process of metastasis of HCC (Hu et al. [25]). Viewed in toto, these genes participate in the progression of HCC, which is consistent with this paper.

Besides, 4 feature genes were not yet well defined in HCC. EIF2S1 catalyzes the first regulatory step in the initiation of protein synthesis to promote the binding of the initial tRNA to the 40S ribosome subunit. Phosphorylated eIF2*α* has been found to predict a triple-negative breast cancer patient's disease-free survival [26]. Estrogen-induced apoptosis of breast cancer cells takes place by blocking dephosphorylation of the eIF2*α* protein [27]. It has been shown that the long noncoding RNA (lncRNA) nR2F1-AS1 stimulates the malignant phenotype of osteosarcoma cells [28]. Inhibition of BIRC5 improves cervical cancer cell sensitivity to radiotherapy [29]. Nine genes, including BIRC5, may be biomarkers for HCC [30]. FKBP1a encodes proteins that are members of the immunomodulatory family, and it is pivotal in immunomodulatory and fundamental cellular processes involved in protein folding and transport. Ten genes, including FKBP1A, were identified as biomarkers for breast cancer [31]. lncRNA SNHG15 enhances EMT of prostate cancer by regulating miR-338-3p/FKBP1A axis [32]. Luo et al. [33] reported FKBP1A overexpression in HCC. Studies have shown that ATG7 adjusts three negative breast cancer tumor progressions [34]. miR-154 exerts a suppressor role by directly targeting ATG7 in bladder cancer [35]. In the context, the investigation of the mechanism of SQSTM1 and HDAC1 in the 6 feature genes was in its infancy. EIF2S1, BIRC5, and FKBP1A were only identified as biomarkers of HCC, and ATG7 was not reported to be associated with HCC. Hence, this paper may provide a theoretic basis for studying these genes in HCC.

On the whole, 6 autophagy-associated genes were identified via bioinformatics methods (EIF2S1, BIRC5, SQSTM1, ATG7, HDAC1, and FKBP1A), and a corresponding prognostic risk model was constructed. Our finding will yield valuable insight into early diagnosis, prognosis, and development of new therapies. However, application of these 6 feature genes requires validation by incremental clinical experiments and animal experiments.

## Figures and Tables

**Figure 1:** Differential expression analysis. (a) Volcano plot of autophagy-related DEGs. Red: differentially upregulated genes; green: differentially downregulated genes; black: gene with no statistical significance. (b) Boxplot of the expression of autophagy-related DEGs. Green: normal tissue; red: tumor tissue.

**Figure 2:** Enrichment analyses of autophagy-related DEGs. (a) GO enrichment analysis. Blue: downregulated; red: upregulated. (b) KEGG enrichment analysis. Blue: downregulated; red: upregulated. The inner circle histogram shows the size of the *p* value. The smaller the *p* value, the higher the column. *Z*-score is defined as the combining expressions of upregulated and downregulated genes. The outer circle shows terms corresponding to the top 10 minimum *p* values.

**Figure 3:** Construction and validation of a prognostic risk model. (a) Forest plot of univariate Cox regression analysis (*p* < 0.0001). (b) Forest plot of multivariate Cox regression analysis. (c) Distribution plot of risk score of patients. (d) Distribution plot of survival status of patients. (e) ROC curves of 3-year and 5-year OS of patients in the training set predicted by 6-gene-based risk model. (f) Kaplan-Meier survival curves of patients in each group in the training set. (g) ROC curves of 3-year and 5-year OS of patients in the validation set predicted by 6-gene risk model. (h) Kaplan-Meier survival curves of patients in each group in the validation set.

**Figure 4:** Risk score with clinical information of TCGA-LIHC patients: (a, b) forest plot of Cox regression analyses; (c) ROC curve of clinical characteristics and risk score.

**Figure 5:** Drawing and validation of the nomogram. (a) 3-year and 5-year OS of HCC patients predicted by the nomogram. (b) Calibration curve of 3-year OS of HCC patients. (c) Calibration curve of 5-year OS of HCC patients.

## Data Availability

The data and materials in the current study are available from the corresponding author on reasonable request.

## Supplementary Materials

Supplementary 1 Supplementary Table 1: clinical information in TCGA-LIHC dataset.

Supplementary 2 Supplementary Table 2: autophagy-related gene data in the Human Autophagy Database.

Supplementary 3 Supplementary Table 3: LIRI-JP in the ICGC database used in this study.
